The article "Construction of Intelligent Nursing System Based on Visual Action Recognition Algorithm" was retracted in 2023. Reasons: unreliable results or conclusions; concerns about the data; concerns about the peer review; concerns about the citations.

# Construction of Intelligent Nursing System Based on Visual Action Recognition Algorithm

**DOI:** 10.1155/2022/8311371

**Published:** 2022-09-20

**Authors:** Yan Zeng, Bo Liang

**Affiliations:** ^1^First Department of Oncology in Yantaishan Hospital, Yantai 264003, China; ^2^Physical Education Department of Shandong Technology and Business University, Yantai 264005, China

## Abstract

Due to advancements in scientific research and technological innovation, as well as the proliferation of the Internet of things, the Internet, and big data, the general public has gradually become aware of a new type of intelligent nursing system model known as the smart nursing system. The smart nursing system is a sensing system and information platform for the elderly in their homes, communities, and institutions for elderly care. Based on this, it provides timely, efficient, and cost-effective elderly care services in real time. These services utilize the Internet of things and the Internet as well. Through the monitoring of video data, we are able to differentiate the visual motions of these elderly individuals and determine whether they are in a normal life state or a fall state. This has the potential to better meet the diverse and multifaceted needs of senior citizens, enhance the quality of life of senior citizens in their final years, and provide senior citizens with greater humanistic care and spiritual solace. Our team has developed an intelligent nursing system based on the visual action recognition algorithm, also known as the deep learning (DL) algorithm. As a result of our simulation tests, we discovered that the algorithm can accurately identify the living situations of elderly individuals at home.

## 1. Introduction

As a result of ongoing advances in medical technology, the medical industry has begun implementing intelligent nursing [1–4] into clinical practice. In addition, the medical industry has created a smart hospital nursing system that combines intelligence, automation, informatization, and digitization to make nursing care more convenient and standardized. To eliminate potential risks posed by human factors, work pertaining to nursing administration is required. By using smart nursing, it is possible to evaluate and care for the physical condition of the elderly at an early stage, thereby reducing the likelihood of accidents and problems and increasing nursing satisfaction. This intelligent nursing system not only increases the efficiency of nursing work [5, 6] and the postoperative efficacy of patients, but it also reduces the cost of medical care.

Seniors have a greater need for attentive care after undergoing a variety of medical procedures in the hospital. Smart nursing encompasses clinical nursing, nursing management, smart medical [7], continuous nursing, and all other nursing-related fields. It focuses on scenarios and regions, employs numerous information technologies (such as cloud computing, the Internet of things, artificial intelligence, large-scale data, etc.), and establishes a platform-based nursing system that is standard, intelligent, and intelligently intelligent. Smart nursing is a relatively new technology, a new concept, and a business model within the profession of nursing. Smart nursing is primarily concerned with integrating nursing activities with information technology platform applications. As a method of nursing administration, the implementation of a smart nursing early warning system based on a visual action recognition algorithm is not only innovative and applicable but also reliable, controllable, effective, and secure.

The article "Construction of Intelligent Nursing System Based on Visual Action Recognition Algorithm" was retracted in 2023. Reasons: unreliable results or conclusions; concerns about the data; concerns about the peer review; concerns about the citations.

Activity recognition [8–13] is an essential component of physical activity monitoring systems and has been the subject of extensive research. There are monitoring systems that utilize sensor devices worn on the body, as well as monitoring systems that can monitor video streams. Some individuals have considered developing activity recognition systems employing small additional sensor chips or wearable sensing devices. Recent research has shown that wearing Google Glass or a bracelet can improve the accuracy of motion detection. There are numerous wearable devices available, including the Apple Watch. They use a variety of sensors to monitor the user's movement and can distinguish between walking, running, and other forms of physical activity. However, their use in continuous monitoring is limited due to high additional costs and stringent restrictions. Given the breadth of sensors that are built into smartphones, activity recognition offers a solution for long-term activity tracking. As smartphone ownership becomes more widespread, the significance of this solution will increase. Vision-based human motion recognition [14–16] is one method for recognizing and analyzing human motion in video captured by a camera. It includes biomechanics, machine vision, image processing, pattern recognition, and artificial intelligence. This is a difficult and multidisciplinary field of study with enormous implications for numerous fields, such as education, business, and society. Human motion recognition is crucial for a wide variety of applications. These applications exist in numerous fields, including robotics, arts and entertainment, sports, medicine, surveillance, content-based video storage and retrieval, human-machine interfaces, and videoconferencing.

The article "Construction of Intelligent Nursing System Based on Visual Action Recognition Algorithm" was retracted in 2023. Reasons: unreliable results or conclusions; concerns about the data; concerns about the peer review; concerns about the citations.

Human action recognition is an important research topic in the field of computer vision, and it has numerous applications in intelligent monitoring, smart homes, and service robots, among others. Computer vision focuses on the analysis of images of the physical world. Due to the development of society, the problem of an aging population is becoming more urgent. As a result, robots that provide household services have been developed. It will continue to attract increasing attention, making full use of home service robots, for example, so that older people's day-to-day needs can be met without placing a burden on younger generations. The core of the technology that powers home service robots is motion recognition. To fulfill their mission of providing care for elderly individuals, these machines must be able to comprehend the intentions of the elderly and respond appropriately. In order to achieve this objective, the challenge of motion recognition will be the first problem to be resolved. In addition, there are numerous literary works based on the recognition of visual actions. Due to its widespread application in the fields of intelligent video surveillance, video retrieval, human-computer interaction, and smart home, video action recognition has become an extremely active area of research in recent years. This is because video action recognition can detect a vast array of human behaviors. Using a method that is considered to be state-of-the-art, positive results have been reported for human action datasets. Local spatiotemporal features and feature bag representations achieve an exceptional level of performance in action recognition when compared to other approaches. A group of researchers first introduced the concept of spatiotemporal interest points [17] by extending the two-dimensional Harris-Laplace detector.

In the third and final section of this report, we discuss the visual action recognition research conducted on the Zhihu nursing system. In the third section, we provide a summary of the data processing techniques and algorithms utilized in our research. In the fourth section, we present the results of our model. In Section 5, we present our conclusions.

## 2. Related Work

There have been significant advancements in the fields of human motion recognition and analysis over the past two decades. As a result, a vast body of literature exists in the form of journals, transaction papers, patents, reviews, and surveys. Tracking the dimensions of the space, the researchers used various types of models (such as stick-based, volumetric, and statistical models) to classify previous work in this area. Several studies have categorized the body of research according to the difficulty of the behaviors that needed to be identified (e.g., gestures, movements, interactions, and group activities). Some studies categorize the current literature based on sensor modality (such as visual, infrared, or range), sensor multiplicity, various applications, number of individuals, number of tracked limbs, and assumptions (such as rigid, nonrigid, or elastic).

The article "Construction of Intelligent Nursing System Based on Visual Action Recognition Algorithm" was retracted in 2023. Reasons: unreliable results or conclusions; concerns about the data; concerns about the peer review; concerns about the citations.

Sensors provide the majority of the information required for human action recognition research [18–20]. There are RGB cameras, Kinect sensors, and wearable inertial sensors among these sensors. Traditional RGB cameras are extremely sensitive to factors such as lighting conditions, background complexity, and partial occlusions when used to capture 2D images. Moreover, the 2D images captured by RGB cameras contain a substantial amount of sensitive information about the subject. Compared to RGB cameras, depth sensors can provide 3D motion data, which are less sensitive to variations in light and illumination levels during acquisition, require fewer resources, and can effectively protect the privacy of the monitored individual. Changes in perspective, noise, and other factors that occur during the process of acquiring depth photographs affect the acquisition's final results. Some researchers use camera movement to correct dense trajectories, extract robust features for acceleration, and use a random sampling consensus algorithm to correct images and eliminate camera movement trajectories to obtain more robust feature descriptors. Additionally, camera motion is used to correct dense trajectories. It is common practice to extract kinematic parameters such as velocity and acceleration when gathering data on dynamics. Using RGB video data, some researchers construct discriminative hierarchical feature representations at different temporal granularities [21, 22]. They then propose a hierarchical sequential summary model for modeling. Some researchers attempt to determine the possible range of joint angle trajectories for the purpose of action recognition, a highly interpretable technique that is used to automatically select the skeleton joint points that can represent the primary information of the current action. The proposed model is known as the major information joint series model.

There are a large number of published works on both action recognition and the design of intelligent nursing systems for the elderly. In the following section, we will discuss the intelligent body care system's construction. The intelligent nursing system employs cutting-edge technology and incorporates findings from extensive research into other intelligent nursing initiatives. It aims to make senior citizens' lives easier and safer, as well as provide them with assistance through the use of technology. It aims to understand the language and facial expressions [23], that is, judge the emotions of the elderly, always detect the health data of the elderly, monitor their health status, and notify the emergency contact promptly when an accident occurs. This safeguards the physical and mental health of the elderly and meets their needs by addressing both their physical and psychological needs. There has been an additional success in intelligent nursing research, including the fact that there is no shortage of intelligent nursing for the elderly. The environmental assisted living system [24] that was just released by the company is designed for senior citizens. Under this system, the elderly will also be able to receive safe geriatric care in the comfort of their own homes and independent living.

The article "Construction of Intelligent Nursing System Based on Visual Action Recognition Algorithm" was retracted in 2023. Reasons: unreliable results or conclusions; concerns about the data; concerns about the peer review; concerns about the citations.

After surgical procedures, nursing, which can be viewed as a form of ongoing therapy, is the primary concern for patients [25]. In addition, continuity of care may involve communication between patients and their providers, individualized care, and the efficient implementation of discharge care programs. When we build a system for intelligent nursing, we will have access to a wealth of information about intelligent nursing. Some academics believe that, from a limited perspective, the purpose of information systems is to collect, further process, and process data in addition to assisting decision-makers from all walks of life. This belief is supported by the vast quantities of data that already exist. According to the opinions of a number of researchers [26], we must share information in order to maximize the utilization of available resources. By implementing this method, it will be possible to enhance the flow of communication between the industry's various departments. In addition, the concept of system management will be applicable to technology, allowing the system to acquire additional technical support for the upcoming work process. Several academics pointed out that in the application of big data, the mixed data itself makes it more difficult for people to make decisions. Because of this, it is easier for users to accept and utilize the analysis results when they are presented in an approachable manner.

## 3. Research Design

### 3.1. Data Sources

The experiment was carried out with the help of the programming language Python and the PyTorch DL framework. Window 8 served as the operating system. The camera on the cell phone was used as the basis for the data collection that was performed.

Six different types of common human motion data, including walking, waving, turning around, picking up, sitting down, and drinking water, were collected from a total of 32 different persons. Every action was repeated thirty times in a free and open setting outside, one after the other. The remaining tasks were accomplished while standing up, except for the one that required sitting down. The acts of picking up and drinking the water were performed with the tester's dominant hand, regardless of whether that was their left or right hand. Each time the data were collected, it was only performed until the end of an entire action, and then that action was reset before the next started so that data could be collected on the following whole action.

The article "Construction of Intelligent Nursing System Based on Visual Action Recognition Algorithm" was retracted in 2023. Reasons: unreliable results or conclusions; concerns about the data; concerns about the peer review; concerns about the citations.

Before the experiment began, all of the gathered files were renamed in accordance with the action name serial number convention. Following this, 85 percent of the files were chosen at random to serve as the training set, and the remaining 15 percent were put to use as the test set. After reading the data from the event stream, batch training was used for training. This meant that throughout the experiment, a batch of training data was entered at a time, which helped speed up the process of training the action recognition network.

### 3.2. CNN Building

GoogLeNet is made up of a deep convolutional neural network design that is known by its secret code name, Inception. This architecture is distinguished by the fact that it enhances the use of computer resources, thereby enhancing the network's overall performance.

#### 3.2.1. Inception Network Architecture

Deep convolutional neural networks, such as Google's GoogLeNet, are created by increasing the depth and breadth of the underlying network model. When attempting to deepen a network, simply increasing the size of the network will result in overfitting and processing issues. In order to resolve this issue, it is necessary to reduce the parameter values while simultaneously increasing the network's depth and width. Due to this, each node in the convolutional neural network must have only a few connections. Due to this, a network architecture for Inception has been developed that is not only capable of sparsely lowering parameters but also of utilizing dense matrix optimization in hardware. The Inception model is presented in Figure 1.

#### 3.2.2. The Human Action Recognition Method Based on GoogLeNet

Figure 2 provides a visual representation of the GoogLeNet model as a whole as it appears in this publication. The convolution and Inception modules are represented by gray, the pooling layer by blue, the fully connected layer by red, the Softmax classification layer by yellow, and the classification output layer by green.

The article "Construction of Intelligent Nursing System Based on Visual Action Recognition Algorithm" was retracted in 2023. Reasons: unreliable results or conclusions; concerns about the data; concerns about the peer review; concerns about the citations.

An extension of the logistic regression classification known as the Softmax regression classification method is utilized in this study in order to better solve the multiclassification problem. This is because the classification of human actions is a multiclassification, that is, mutually exclusive.

If we assume that there are *I* categories involved in the multiclassification problem, then *y*^*k*^ ∈ {1,2, *i*}. In the method of Softmax regression, the hypothesis function calculates, for any given test *x*, an estimate of the likelihood of each class appears as

(1) $$\begin{array}{c} c_{\alpha }\left(x^{k}\right)=\left(\begin{array}{c} p\left(y^{k}=1|x^{k};\alpha \right)\\ p\left(y^{k}=2|x^{k};\alpha \right)\\ ...\\ p\left(y^{k}=i|x^{k};\alpha \right) \end{array}\right)=\frac{1}{\overset{i}{\underset{h=1}{\sum }}e^{\alpha_{h}^{R}x^{k}}}\left(\begin{array}{c} e^{\alpha_{1}^{R}x^{k}}\\ e^{\alpha_{2}^{R}x^{k}}\\ ...\\ e^{\alpha_{i}^{R}x^{k}} \end{array}\right)\text{.} \end{array}$$

Each row of the matrix is considered to represent a category that corresponds to the parameters of the classifier. This results in the model parameter *α* being transformed into a matrix that has a total of *I* rows. It is possible to write the matrix *α* in the following form:

(2) $$\begin{array}{c} \alpha =\left(\begin{array}{c} \alpha_{1}^{R}\\ \alpha_{2}^{R}\\ ...\\ \alpha_{i}^{R} \end{array}\right)\text{.} \end{array}$$

The normalization of the probability distribution is denoted by the symbol ∑_*h*=1_^*i*^*e*^*α*_*h*_^*R*^*x*^*k*^^ in formula (1), and its function is to ensure that the aggregate of all probabilities is equal to 1.

In the same vein, the equation for the system's loss function can be written as

(3) $$\begin{array}{c} E\left(\alpha \right)=-\frac{1}{b}\left[\overset{b}{\underset{k=1}{\sum }}\overset{i}{\underset{h=1}{\sum }}I\left\{y^{k}=h\right\}\log\frac{e^{\alpha_{d}^{R}x^{k}}}{\overset{i}{\underset{d=1}{\sum }}e^{\alpha_{d}^{R}x^{k}}}\right]\text{.} \end{array}$$

In the formula, *I*{·} acts as an indicator function, and the value rule is that I{expression with true value} = 1, *I*{expression with false value} = 0.

The probabilities of *I* categories are tallied up by the Softmax regression classification method, and the likelihood that the *x* category is in fact the *j* category is calculated as the product of those two numbers.

(4) $$\begin{array}{c} p\left(y^{k}=j|x^{k};\alpha \right)=\frac{e^{\alpha_{j}^{R}x^{k}}}{\overset{i}{\underset{j=1}{\sum }}e^{\alpha_{j}^{R}x^{k}}}\text{.} \end{array}$$

A generalization of the loss function used in logistic regression is represented by equation (3). The loss function of the model can also be represented as shown, which can be used to minimize the model parameter *α*.

(5) $$\begin{array}{c} \begin{array}{c} E\left(\alpha \right)=-\frac{1}{b}\left[\overset{b}{\underset{k=1}{\sum }}y^{k}\;\log c_{\alpha }\left(x^{k}\right)+\left(1-y^{k}\right)\log\;\left(1-c_{\alpha }\left(x^{k}\right)\right)\right]\\ =-\frac{1}{b}\left[\overset{b}{\underset{k=1}{\sum }}\overset{d}{\underset{j}{\sum }}I\left\{y^{k}=j\right\}\log\;p\left(y^{k}=j|x^{k};\alpha \right)\right] \end{array}\text{.} \end{array}$$

When performing multiclass recognition, the loss function must also be minimized; an iterative optimization technique, such as gradient descent, is typically employed for this purpose.

The article "Construction of Intelligent Nursing System Based on Visual Action Recognition Algorithm" was retracted in 2023. Reasons: unreliable results or conclusions; concerns about the data; concerns about the peer review; concerns about the citations.

The initial step of the gradient descent method is to calculate the partial derivative of the loss function.

(6) $$\begin{array}{c} \nabla_{\alpha_{j}}E\left(\alpha \right)=-\frac{1}{b}\overset{b}{\underset{k=1}{\sum }}\left[x^{k}\left(I\left\{y^{k}=j\right\}-p\left(y^{k}=j|x^{k};\alpha \right)\right)\right]\text{,} \end{array}$$

where ∇_*α*_*j*__*E*(*α*) is a vector and each of its components, *∂E*(*α*)/*∂α*_*jl*_, represents a partial derivative of the loss function with respect to the *i*th parameter of *j* categories. In the gradient descent algorithm, equation (6) is substituted, and after each iteration, the iterative is updated *α*_*j*_=*α*_*j*_ − *β*∇_*α*_*j*__*E*(*α*)(*j*=1,2, *i*) to determine the loss function that is minimized.

When the aforementioned functions are utilized directly in the classification process using Softmax regression, there will be redundant parameter sets. This will have an influence on the way that updates are performed on parameters. As a result, the loss function will be adjusted as described below:

(7) $$\begin{array}{c} p\left(y^{k}=j|x^{k};\alpha \right)=\frac{e^{\left(\alpha_{j}-\phi \right)R_{x^{k}}}}{\overset{i}{\underset{l=1}{\sum }}e^{\left(\alpha_{l}-\phi \right)R_{x^{k}}}}=\frac{e^{\alpha_{j}R_{x^{k}}}}{\overset{i}{\underset{l=1}{\sum }}e^{\alpha_{l}R_{x^{k}}}}\text{.} \end{array}$$

According to equation (7), the value of the loss function that is derived by deducting the same value from each item of the obtained optimization parameter does not vary, which demonstrates that this parameter is not the only answer to the problem. The weight decay term *μ*/2∑_*k*=1_^*i*^∑_*j*=0_^*m*^*α*_*kj*_^2^ is added to the loss function during the design phase of the classification in order to address the issue brought about by the fact that the parameters do not have a unique value global optimal solution. When we reach this stage, the loss function transforms into

(8) $$\begin{array}{c} E\left(\alpha \right)=-\frac{1}{b}\left[\overset{b}{\underset{k=1}{\sum }}\overset{i}{\underset{j=1}{\sum }}I\left\{y^{i}=j\right\}\log\frac{e^{\alpha_{j}R_{x^{k}}}}{\overset{i}{\underset{i=1}{\sum }}e^{\alpha_{i}R_{x^{k}}}}\right]+\frac{\mu }{2}\overset{i}{\underset{k=1}{\sum }}\overset{m}{\underset{j=0}{\sum }}\alpha_{kj}^{2}\text{,} \end{array}$$

where *μ* > 0. The expression of the loss function using the partial derivative function is as follows:

(9) $$\begin{array}{c} \nabla_{\alpha_{j}}E\left(\alpha \right)=-\frac{1}{b}\overset{b}{\underset{k=1}{\sum }}\left[x^{k}\left(I\left\{y^{k}=j\right\}-p\left(y^{k}=j|x^{k};\alpha \right)\right)\right]+\mu \alpha_{j}\text{.} \end{array}$$

After everything was said and done, the minimized loss function and the Softmax regression classification model were finally obtained.

The article "Construction of Intelligent Nursing System Based on Visual Action Recognition Algorithm" was retracted in 2023. Reasons: unreliable results or conclusions; concerns about the data; concerns about the peer review; concerns about the citations.

In this study, the multiclassification problem of actions is addressed using the Softmax classification, which is a type of logical classification. This classification is employed in the classification of this model. Because the database being accessed contains 6 different sorts of operations, the value of *i* is 6. In addition to this, it is validated by the development of an action recognition model application system.

As can be seen from the table, the accuracy rate serves as the evaluation index for the model.

(10) $$\begin{array}{c} Acc=\frac{TP}{TP+FN+FP+TN}\text{.} \end{array}$$

#### 3.2.3. Output Layer Visualization

The purpose of the visualization of the output layer is to establish a connection between the recently added classification output layer and the established action recognition model application system. This is performed in order to facilitate the display of the input image discrimination process in the form of a graphical user interface for MATLAB.

## 4. Results

Comparing the convolutional neural network algorithm (CNN) with the multilayer perceptron algorithm (MLP), which are both algorithms, results in the name OUR algorithm being given to the GoogLeNet method.

As depicted in Figure 3, the precision attained by each of the three algorithms varies as a function of the total number of iterations. The evaluation index of accuracy reveals that the OUR algorithm, the CNN algorithm, and the MLP algorithm all achieved positive experimental outcomes. This demonstrates that the three methods can be successfully applied to the field of visual action recognition-based intelligent nursing system construction. In addition, it is evident from the figure that in the three groups of human action recognition experiments, the OUR algorithm exhibits an improvement in the evaluation index of accuracy, demonstrating its superiority. This is evidenced by the fact that the evaluation index of accuracy for the OUR algorithm is significantly higher than that for the CNN algorithm and the MLP algorithm.

The article "Construction of Intelligent Nursing System Based on Visual Action Recognition Algorithm" was retracted in 2023. Reasons: unreliable results or conclusions; concerns about the data; concerns about the peer review; concerns about the citations.

As shown in Figure 4, the loss value of each of the three methods varies based on the number of iterations. As the number of iterations increases, it is evident that the respective losses of the three algorithms decrease linearly. When the number of iterations reaches approximately 180, the reduction rate produced by the OUR algorithm tends to stabilize. The CNN algorithm reaches a stable state when the number of iterations reaches approximately 200. When the number of iterations reaches approximately 140, the loss value produced by the MLP algorithm tends to settle into a steady state. When the final loss values of the three algorithms are compared, it is found that the OUR algorithm has the lowest loss value, followed by the CNN algorithm, and the MLP algorithm has the highest loss value.

Figure 5 depicts the results of a comparison of the time required to execute each of the three algorithms during the experimental simulation. It is evident that the MLP method has the quickest running time, followed by the OUR algorithm and finally by the CNN algorithm, which has the slowest running time. The structure of the three algorithms suggests that the model parameters of the OUR algorithm are greater than those of the MLP algorithm; thus, the time required for the OUR algorithm to complete its task is longer than the time required for the MLP algorithm to complete its task.

The results of a comparison of the three algorithms' recall and precision rates are presented in Table 1. We can see that when we compare the performance of the three algorithms using these two evaluation indicators, we can see that the precision and recall rates of the OUR algorithm are higher than those of the CNN algorithm and the MLP algorithm. This is something that we can see when we compare the performances of the three algorithms.

## 5. Conclusion

The construction of a smart nursing system that is based on visual action recognition algorithms to improve the service quality, service level, and service efficiency of healthy elderly care services is not only a choice against the backdrop of China's aging population but also a crucial component of the healthy China strategy. This system aims to improve the service quality, service level, and service efficiency of services for healthy elderly care. Despite this, the industry of intelligent care for the elderly in the country is still in its infancy, and there are numerous obstacles on both the technological and application fronts. This research constructs an intelligent nursing system using a visual action recognition algorithm and a deep learning algorithm. This system is capable of identifying activities in various application scenarios, performing analysis, and issuing alerts to compensate for the fragmentation of traditional smart elderly care product scenarios. It has the potential to effectively protect the health and well-being of senior citizens in their communities of residence. Within the context of the new era, the issue of elderly care has garnered significant attention, and it has become a crucial obligation to provide a better environment and services for the elderly.

The article "Construction of Intelligent Nursing System Based on Visual Action Recognition Algorithm" was retracted in 2023. Reasons: unreliable results or conclusions; concerns about the data; concerns about the peer review; concerns about the citations.

The purpose of this study is to make a proposal for the development of an intelligent nursing system based on an algorithm that has been successfully applied to the field of human action recognition for the recognition of visual actions. The results of these experiments indicate that the methodology presented in this study is capable of discriminating precisely between six distinct action postures. This method not only presents a novel research concept for the fields of DL and human action recognition but also provides a novel research reference for the fields of rehabilitation exercise and physical training. Using this methodology will benefit both of these fields of study. There is a chance that interference will occur throughout the experiment. Therefore, it is advised that this experiment be conducted in an area devoid of interference.

## Figures and Tables

**Figure 1:** Inception model.

**Figure 2:** Improved overall structure of GoogLeNet.

**Figure 3:** Accuracy as a function of the number of iterations.

**Figure 4:** Loss values under different models.

**Figure 5:** Runtime under different models.

**Table 1:** Precision and recall of the three algorithms.

	Precision (%)	Recall (%)
OUR	89.36	87.63
CNN	86.58	86.54
MLP	87.69	83.28

## Data Availability

The data used to support the findings of this study are available from the corresponding author upon request.

## References

[1] Six smith A., Six smith J. (2000). Smart care technologies: meeting whose needs?. *Journal of Telemedicine and Telecare*.

[2] Poncela A., Coslado F., García B. (2019). Smart care home system: a platform for E-Assistance. *Journal of Ambient Intelligence and Humanized Computing*.

[3] Hong Y. S. (2018). Smart care beds for elderly patients with impaired mobility. *Wireless Communications and Mobile Computing*.

[4] Thomas A. M., Moore P., Shah H. (2013). Smart care spaces: needs for intelligent at-home care. *International Journal of Space-Based and Situated Computing*.

[5] Brooks B. A., Anderson M. A. (2005). Defining quality of nursing work life. *Nursing Economics*.

[6] Upenieks V. V. (1998). Work sampling: assessing nursing efficiency. *Nursing Management*.

The article "Construction of Intelligent Nursing System Based on Visual Action Recognition Algorithm" was retracted in 2023. Reasons: unreliable results or conclusions; concerns about the data; concerns about the peer review; concerns about the citations.

[7] Winter A., Stäubert S., Ammon D. (2018). Smart medical information technology for healthcare (SMITH). *Methods of Information in Medicine*.

[8] Kim E., Helal S., Cook D. (2010). Human activity recognition and pattern discovery. *IEEE pervasive computing*.

[9] Chen L., Hoey J., Nugent C. D., Cook D. J., Yu Z. (2012). Sensor-based activity recognition. *IEEE Transactions on Systems, Man, and Cybernetics, Part C (Applications and Reviews)*.

[10] Huynh T., Schiele B. Analyzing features for activity recognition.

[11] Vrigkas M., Nikou C., Kakadiaris I. A. (2015). A review of human activity recognition methods. *Frontiers in Robotics and AI*.

[12] Ravi N., Dandekar N., Mysore P., Littman M. L. (2005). Activity recognition from accelerometer data. *Aaai*.

[13] Ke S. R., Thuc H. L. U., Lee Y. J., Hwang J. N., Yoo J. H., Choi K. H (2013). A review on video-based human activity recognition. *Computers*.

[14] Kale G. V., Patil V. H. (2016). A study of vision based human motion recognition and analysis[J]. *International Journal of Ambient Computing and Intelligence*.

[15] Poppe R. (2007). Vision-based human motion analysis: an overview. *Computer Vision and Image Understanding*.

[16] Moeslund T. B., Hilton A., Krüger V. (2006). A survey of advances in vision-based human motion capture and analysis. *Computer Vision and Image Understanding*.

[17] Zhou T. A scale invariant keypoints detector.

[18] Chu X., Kobialka T., Durnota B., Buyya D. Open sensor web architecture: core services.

[19] Aggarwal C. C. (2013). *Managing and Mining Sensor data*.

[20] Tham C. K., Buyya R. (2005). SensorGrid: integrating sensor networks and grid computing. *CSI Communications*.

[21] Liu L., Shao L. Learning discriminative representations from RGB-D video data.

[22] Yu M., Liu L., Shao L. (2016). Structure-preserving binary representations for RGB-D action recognition. *IEEE Transactions on Pattern Analysis and Machine Intelligence*.

[23] Özer D., Göksun T., Chatterjee A. (2019). Differential roles of gestures on spatial language in neurotypical elderly adults and individuals with focal brain injury. *Cognitive Neuropsychology*.

[24] Sun H., De Florio V., Gui N., Blondia C. Promises and challenges of ambient assisted living systems.

[25] Kennedy E. H., Ma Z., McHugh M. D., Small D. S. (2017). Non‐parametric methods for doubly robust estimation of continuous treatment effects. *Journal of the Royal Statistical Society: Series B*.

[26] Longo D. L., Drazen J. M. (2016). Data sharing. *New England Journal of Medicine*.

